# Influence of a fully magnetically levitated left ventricular assist device on functional interrogation of implantable cardioverter defibrillators

**DOI:** 10.1002/clc.23228

**Published:** 2019-07-07

**Authors:** Christoph Schukro, Thomas Schlöglhofer, Cesar Khazen, Michael Röhrich, Günther Laufer, Daniel Zimpfer, Dominik Wiedemann

**Affiliations:** ^1^ Department of Internal Medicine II, Division of Cardiology Medical University of Vienna Vienna Austria; ^2^ Department of Surgery, Division of Cardiac Surgery Medical University of Vienna Vienna Austria; ^3^ Department of Anesthesia, Intensive Care Medicine and Pain Therapy Medical University of Vienna Vienna Austria; ^4^ Ludwig‐Boltzmann‐Cluster for Cardiovascular Research Vienna Austria

**Keywords:** impaired interrogation, implantable cardioverter defibrillator, interference, left ventricular assist device

## Abstract

**Background:**

Electromagnetic interference between left ventricular assist devices (LVAD) and the telemetry wand of implantable cardioverter‐defibrillators (ICD) with impairment of ICD interrogation has previously been described in *HVAD* and *HeartMate II* devices. This is the first study showing the potential influence of the LVAD model *HeartMate 3* (with the unique feature of fully magnetically levitated rotor with consistent wide blood‐flow gaps) on functional interrogation of different ICD models.

**Methods and Results:**

Among 51 patients treated with a *HeartMate 3* LVAD, 34 patients (66.7%) already had an ICD implanted prior to LVAD therapy. In this cohort, impairment of ICD interrogation was observed in five patients (14.7%) with five different device models. In patients with *Biotronik* ICD, stretching of the ipsilateral arm to increase the distance between both devices >10 cm was sufficient in one patients, whereas surgical contralateral repositioning was necessary in two patients; in one further patient no action could be taken, as he died early from embolic stroke. In the only patient with a *MicroPort* ICD, this issue was resolved by using a wireless telemetry. The distances between both devices showed no statistical significant correlation with an impaired interrogation, neither in the overall collective nor within the groups with the same manufacturer.

**Conclusions:**

In patients with impaired ICD interrogation caused by electromagnetic interference between a *HeartMate 3* LVAD and the ICD, the actions mentioned above have to be taken, to resolve this technical issue. Especially, a sufficient distance of at least 10 cm between both devices was crucial for avoiding this problem.

## 1 INTRODUCTION

Left ventricular assist devices (LVAD) are increasingly used as bridge to heart transplantation and destination therapy in patients with end‐stage congestive heart failure.^1^ The *HeartMate 3* LVAD (Abbott Laboratories, Abbott Park, Illinois) received the European Conformity mark October 2, 2015 2 and was implanted already in more than 1000 patients.^3^ The unique feature of this continuous flow LVAD is the fully magnetically levitated rotor with consistent wide blood‐flow gaps designed to reduce shear stress on blood components and to enhance biocompatibility (Figure 1).

**Figure 1:** Schematic depiction of *HeartMate 3*

Low static electromagnetic fields of 0.1 T are known to affect the functional interrogation of implantable cardiac devices, that is, cardiac pacemakers or implantable cardioverter‐defibrillators (ICD). 3 Furthermore, specific magnets—in the form of either doughnuts or bars— with a slightly lower static magnetic field strength of almost 0.05 T are widely used for temporary deactivation of the anti‐tachycardia function of an ICD, for example, during electrocautery.

The following study is the first to report on the potential influence of the LVAD model *HeartMate 3* on functional interrogation of different ICD models.

## 2 METHODS

### 2.1 Patient population

In this retrospective, single‐center study, 51 patients were analyzed after implantation of a *HeartMate 3* LVAD between June 2014 and September 2017 at the Medical University of Vienna, Austria. The mean age was 62.4 ± 8.9 years, 88.2% were male, with an average body mass index (BMI) of 28.2 ± 5.1 kg/m^2^. Twenty‐eight of our 51 patients (54.9%) had ischemic cardiomyopathy, as diagnosed by coronary angiography in all cases. At the time of implantation, 21.6% were in INTERMACS profile 1, 15.7% profile 2, 17.6% profile 3, 45.2 profiles 4 to 7.

Among our 51 patients, overall 34 (66.7%) had already an ICD implanted prior to the LVAD therapy, all of them for primary prevention of sudden cardiac death.

ICD devices of five different manufacturers were implanted: Biotronik (Berlin, Germany) in 11 patients, Medtronic (Dublin, Ireland) in 10 patients, Abott Laboratories (formerly St. Jude Medical) in 7 patients, MicroPort (formerly Sorin or LivaNova; Shanghai, China) and Boston Scientific (Marlborough, Massachusetts) in three patients each.

### 2.2 Technical issue

In this cohort, we incidentally found an impaired functional ICD interrogation in five patients. In other words, in these patients the technical device interrogation was either completely or partially disabled (details are presented in the Section 3). In the other 29 patients, such impairment was not observed at all. Therefore, ICD types, extent of interference with *HeartMate 3*, as well as problem solving strategies were retrospectively analyzed.

### 2.3 Measurement of distance

Whenever applicable, frontal and lateral chest X‐ray images (DICOM format) were used for measurements of distance between ICD and *HeartMate 3*. As shown in Figure 2 *,* the shortest distance was measured between the edges of both devices, using the ImageJ software.

**Figure 2:** Measurement of distance between implantable cardioverter‐defibrillator and *HeartMate 3*

### 2.4 Statistics

The statistical analysis was performed using SPSS for Windows Release 23.0.0 (SPSS Inc. Chicago, Illinois). Metric variables are reported as mean ± SD (SD) for normally distributed data or as the median with the interquartile range (IQR) for non‐normally distributed data, and compared with Student's *t* test of Mann‐Whitney test, respectively. Normal distribution was assessed by the Shapiro‐Wilk test. One‐way analysis of variance (ANOVA) followed by post hoc comparison with Bonferroni correction was employed to determine statistical significance levels among the 5 ICD manufacturer groups. Statistical significance was considered at *P* < .05.

## 3 RESULTS

Among our collective of 34 *HeartMate 3* patients with an active ICD therapy, functional interrogation of the ICD device remained unsuccessful in five patients (14.7%). In all the other patients with an unimpaired ICD interrogation, no technical problems regarding function parameters, battery voltage or inappropriate noise‐artifact detection were documented.

In four patients with devices of the manufacturer *Biotronik*, the electromagnetic interference between the magnetic LVAD motor and the telemetry wand made the interrogation of the ICD completely impossible, that is, the programmer monitor remained in the “start screen” as no communication could be built between the ICD and the programmer. In two of these patients *(devices: Iforia HF‐T with 3 leads, and Itrevia VR‐T with 1 lead)*, the device was surgically repositioned contra‐laterally to interrogate and program the ICD system. The first of these patients showed one episode of appropriate anti‐tachycardia pacing for ventricular tachycardia (VT) and two appropriate shocks for ventricular fibrillation; the second got one appropriate shock for a fast VT. All these appropriate interventions were successful. In one further patient (*device: Itrevia DR‐T with two leads*), stretching of the ipsilateral (left) arm enabled the interrogation by increasing the distance between the two devices. Once device interrogation was enabled, we found no technical issue regarding function parameters, battery voltage or inappropriate artifact detection in these patients.

The fourth of these patients (*device: Lumax VR‐T with one lead*) got multiple appropriate shocks for ventricular fibrillation while on continuous intensive care monitoring, but died early because of a multifocal embolic stroke after myocardium suction by the LVAD, before any specific action could be taken regarding the ICD position.

In one further patient with an ICD including cardiac resynchronization therapy function of the manufacturer *MicroPort* (*device: Platinum SonR CRT‐D*) only the initial interrogation screen with a persisting “interrogating” signal was displayed, but no further functional testing or programming were possible. Thus, we had information about automatically measured lead impedances and sensing (both parameters were normal), but no pacing‐threshold testing or battery voltage measurement could be performed. Remarkably, the complete “offline” information about the ICD system could be interrogated afterwards. In this special case, the interrogation of the ICD could be performed in the following visits by a special wireless telemetry, which has a higher data transfer rate than the standard telemetry wand. Afterwards, this patient showed no technical issues as well.

Remarkably, the manually measured distances between both devices showed no statistical significant correlation with an impaired ICD interrogation in both planes, neither in the overall collective (impairment vs no impairment in the lateral plane: 107.0 ± 17.6 mm vs 94.8 ± 33.9 mm, *P* = .487, as well as in the frontal plane: 68.2 ± 29.0 mm vs 49.1 ± 31.8 mm, *P* = .517) nor within the groups of patients with the same manufacturer (for homogenous subsets in lateral plane: *P* = .458, and in frontal plane: *P* = .606). In patients with *Biotronik* devices, ICD with impaired interrogation were located closer to the LVAD than those without interactions, although not significantly (lateral: 100.0 ± 19.1 mm vs 111.0 ± 38.7 mm, *P* = .352; frontal: 54.0 ± 11.0 mm vs 67.0 ± 38.1 mm, *P* = .560).

## 4 DISCUSSION

To date, there are a few published reports of negative interactions between ICD and LVAD devices other than the *HeartMate 3*. Two case reports^4^, ^5^ of patients with an interaction between ICD and *HeartMate II* LVAD were described, that resulted in an inability to interrogate and program the ICD, ultimately requiring replacement of the ICD. Additionally, two reports on inappropriate ICD shocks^6^, ^7^ and one report with pacing inhibition^8^ in patients with Medtronic HVAD device were reported.

To the best of our knowledge, this is the first series on impaired ICD interrogations of multiple device models due to electromagnetic interference between the magnetic motor of the LVAD model *HeartMate 3* and the ICD telemetry wand. This phenomenon has previously been reported in patients with pacemaker or ICD during electrophysiological interventions in a remote magnetic navigation system.^9^

As three of our five patients got successful appropriate ICD interventions (anti‐tachycardia pacing or shocks) for ventricular tachyarrhythmia, the interference obviously concerned only the interrogation, but not the ICD function itself. In our cohort, the technical issue was mainly found in patients with ICD of the company of *Biotronik,* regardless of the device model and the number of connected leads. Remarkably, the same company is the only one where the application of a “bar magnet” on the device is preferred over a “doughnut magnet,” to deactivate temporary the anti‐tachycardia function of the ICD. This circumstance might be a potential explanation for this company‐related technical interference. But, on the other hand, this issue has been found in one patient with an ICD device of the company of *MicroPort*. This fact rather supports the theory of an electromagnetic interference based on the different company‐specific radiofrequencies for device connectivity of the interrogation wand.

Because of the electromagnetic field of the *HeartMate 3* motor with potential influence on the telemetry or on the ICD itself, this issue has been anticipated by the LVAD manufacturer. Thus, the following recommendation is stated in the *HeartMate 3* user's manual regarding the distance between any ICD and this specific LVAD model: “Prior to implanting an implantable cardiac defibrillator or implantable pacemaker in a *HeartMate 3* patient, the device to be implanted should be placed in close proximity to the Pump (approximately 10 cm) and the telemetry verified.”

Although the biplane measured distances between both devices showed no statistically significant correlation with an impaired interrogation (which is explained by the retrospective nature of our analysis and the small sample size), intentional increasing of the distance between the ICD and the *HeartMate 3* LVAD was the most efficient intervention to enable the ICD interrogation in most of the patients.

Therefore, we recommend the following four actions to enable an interrogation in patients with already implanted ICD systems:

1. Stretching the patient's ipsilateral arm, preferably in an upright position, may increase the distance between the two devices to allow an unhindered functional interrogation of the ICD. Of note, this simple action may depend on the actual anatomical position of the device and the patient's height.
2. Using a company‐specific wireless telemetry system whenever applicable (eg, in *MicroPort* devices).
3. Using wireless remote monitoring (eg, *Home Monitoring* in case of a *Biotronik* system) allows at least an interrogation of the most important functional parameters. In this case, there is usually no possibility to program the ICD.
4. If the previous recommendations are not successful, surgical reposition on the contra‐lateral side is the last, but most effective option *(*Figure 3: Distance between ICD and LVAD was 49 mm before and 190 mm after repositioning).

**Figure 3:** Contralateral repositioning of implantable cardioverter‐defibrillator in a patient with *HeartMate 3*

As this study is a retrospective observational analysis in a comparably small collective, further investigations will be necessary to explain the origin of this specific electromagnetic interference of ICDs with the *HeartMate 3* LVAD.

## 5 CONCLUSIONS

In our LVAD cohort, the electromagnetic interference between the *HeartMate 3* LVAD and the telemetry wand interrupted the interrogation of the ICD system. In LVAD candidates with already implanted ICD device, this potential technical problem has to be considered before implantation. In patients with *HeartMate 3* LVAD with the decision to implant an ICD, we recommend to take care of a sufficient distance of at least 10 cm between the two devices.

## CONFLICT OF INTEREST

Thomas Schlöglhofer, Daniel Zimpfer, and Dominik Wiedemann declare consultant contracts and speaker fees for two LVAD producing companies, Abbott and Medtronic, whereas the other authors have no conflict of interest to declare.
